# Kinetics and soft computing evaluation of Linseed oil transesterification via CD-BaCl-IL catalyst

**DOI:** 10.1016/j.heliyon.2024.e37686

**Published:** 2024-09-12

**Authors:** Kenechi Nwosu-Obieogu, Ude Callistus Nonso, Onukwuli Dominic Okechukwu, Ezeugo Joseph

**Affiliations:** a Department of Chemical Engineering, Michael Okpara University of Agriculture, Umudike, Nigeria; b Department of Chemical Engineering, Nnamdi Azikiwe University Awka, Nigeria; c Department of Chemical Engineering, Chukwuemeka Odumegwu University, Uli, Nigeria

**Keywords:** Biodiesel, Linseed oil, Langmuir-Hinshelwood-Hougen-Watson, Eley-Rideal, Clay, Catalyst

## Abstract

A novel clay-doped ionic liquid and BaCl (CD-BaCl-IL) heterogeneous catalyst for biodiesel synthesis from linseed oil (LSO) was generated after 4 h of calcination at 600°C using Scanning Electron Micrograph (SEM), X-ray Diffraction (XRD), Brunauer-Emmett-Teller (BET), Fourier Transform Infrared Spectroscopy (FT-IR) and X-ray fluorescence (XRF) was used to evaluate the catalyst's processability. After optimization using response surface methodology (RSM), the second-order polynomial model was shown in the Analysis of variance (ANOVA) with R^2^ values of 0.9947, Adj R^2^ (0.9850), and Pred R^2^ (0.8594), demonstrating model acceptability. The maximum biodiesel yield (97.097 %) was obtained with 2.6 wt% catalyst, 6 mol/mol methanol/molar ratio, 1.5 h, 50 °C, and 400 rpm agitation. ANFIS predicted biodiesel yield more accurately than ANN (R^2^ = 0.999, MSE = 0.27594), with the lowest MSE (R^2^ = 0.99, MSE = 0.00038). Under optimal conditions, this study employed a kinetic model based on two elementary chemical processes: Eley-Rideal (ER) and Langmuir-Hinshelwood-Hougen-Watson (LHHW). The LHHW model accurately described CD-BaCl-IL catalyst experimental data at 50 °C, with favourable parameters, an R^2^ value of 0.9348, and a variance of 2.61E-8. The surface reaction between adsorbed triglyceride and alcohol dictated the rate-determining step. Temperature increased the rate, indicating an endothermic process. The reaction's activation energy and frequency factor were 10.22 kJ/mol and 6.41 h-1, respectively. Linseed biodiesel met the D6751 criterion.

## List of symbols and abbreviations

ANN: Artificial neural network
ANFIS: Adaptive neuro-fuzzy inference system
ASTM: American Society for Testing and Materials
CCD: Central composite design
CD-BaCl-IL: Clay doped barium cloride/ionic liquid
Ea: Activation energy
FAME: Fatty acid methyl ester
FFA: Free fatty acid
LSO: Linseed oil
SEM: Scanning Electron Micrograph
XRD: X-ray Diffraction
BET: Brunauer-Emmett-Teller
FT-IR: Fourier Transform Infrared Spectroscopy
XRF: X-ray fluorescence
LHHW: Langmuir-Hinshelwood-Hougen-Watson
ER: Eley-Rideal
MLP: Multiplayer perceptron
MSE: Mean square error
RPM: Revolution per minute
RSM: Response surface methodology
ΔH =: Change in enthalpy
ΔS =: Change in entropy
$k_{f}$ =: Forward rate constants
$k_{b}$ =: Backward rate constants
$K_{1},K_{2},K_{3},K_{4},K_{5},K_{6},K_{7},K_{8},K_{9}$ =: Equilibrium constants

## 1 Introduction

Biodiesel, which is produced through vegetable and animal fat transesterification with the help of a catalyst, is considered a more sustainable alternative to petrodiesel [1]. While a homogeneous catalyst is typically faster and more efficient in terms of conversion rates, it presents certain challenges, such as the need for catalyst separation, removal of by-products, and the formation of soap during the reaction due to the high content of free fatty acids (FFA) [[2], [3], [4], [5]]. These challenges can be addressed by using a heterogeneous catalyst [[6], [7], [8], [9]]. Various techniques involving heterogeneous catalysis offer advantages such as reduced production costs, as they make use of renewable materials for the majority of their raw materials, and the ability to be reused [4].

Linseed oil is derived from matured seeds of the flax plant, which belongs to the Linaceae family [10]. The main countries where flaxseed is grown are China, India, Ethiopia, and the USA with a total world production of 2.65 million tonnes per year. The oil is obtained through solvent extraction and can undergo polymerization, resulting in a solid state [11]. It contains a significant amount of polyunsaturated triglycerides, making it suitable for biodiesel synthesis. Linseed oil has been evaluated as a potential source of biodiesel and confirmed that it exhibited petrodiesel-like characteristics [12] also, the physicochemical characteristics complied with the standards established by ASTM [13].

Clay possesses exceptional catalytic activity due to its porous structure, which allows for the initiation of reactions and facilitates specific molecular interactions, leveraging its inherent qualities [14]. It contains clay minerals, which contribute to its physical characteristics such as rheological properties, ion exchange, swelling, hydration, and plasticity [15]. These materials are inexpensive, abundant, and crucial [16]. According to Abdelkareem and Olabi [17], they exhibit strong thermal stability and can be reused in the transesterification process.

Several researchers have extensively studied the catalytic properties of clay in the transesterification procedure. An alkaline clay catalyst was utilised successfully for gmelina oil transesterification [18]. Salmasi et al. [16] created a catalyst by applying K_2_CO_3_ onto clay to facilitate sunflower oil transesterification, and a biodiesel yield of 98.4 % was obtained. Inayat et al. [15] enhanced the production of biodiesel to 93.6 % from waste frying oil by employing clay as a catalyst. Jalalmanesh et al. [14] produced a biodiesel yield of 95.3 % from sunflower oil by utilising a kaolin catalyst doped with K_2_CO_3_. Through their experiments, it was discovered that clay exhibits remarkable catalytic characteristics during transesterification in maximizing the biodiesel yield.

Researchers can exploit the distinct properties of a material by introducing doping with another chemical [19]. Multiple investigations have recorded the utilisation of doped catalysts, specifically the Zn-doped CaO catalyst, in the transesterification procedure of *Calophylum phylum* oil [20]. The transesterification of canola oil is performed using a catalyst consisting of Na-K impregnated with CaO generated from eggshell [20]. On the other hand, the transesterification of waste oil is carried out using a catalyst called ZnCuO/N-doped nanocatalyst [21]. Their study showcased that the catalyst, when doped, augmented its efficacy by transforming low-grade oils into biodiesel and amplifying the production of biodiesel.

Barium chloride (BaCl) and ionic liquid are selected for doping with clay due to their outstanding catalytic activity, stability, and quick reaction times [22]. Ionic liquids make conducting reactions with higher selectivity and yields possible; however, their most important asset is easy isolation from the catalyst mixture [22]. The use of ILs reduces *the reaction and purification steps. It increases the economic feasibility* and could be one of the advantages of biodiesel production *as low consumption of methanol reduces the production cost* [23,24]*.* However, there are challenges associated with the practical application of ionic liquids in this context, such as their high cost and potential toxicity [24]. Researchers have explored the possibility of doping ionic liquids with clay to address these challenges. Doping ionic liquids with clay can enhance their catalytic properties and stability, making them more suitable for biodiesel production Yusuff et al. [23] obtained a methyl ester yield of 93.17 % by employing a zeolite that underwent barium treatment to carry out transesterification of used frying oil. Dadhnaia et al. [24] conducted a study where they synthesized an ionic liquid utilising a separable heteropolyanion and assessed its catalytic potential for esterifying long-chain fatty acids. Additionally, they examined the impact of several experimental variables, such as the quantity of catalyst, the molar ratio of alcohol to acid, the duration of the reaction, and the temperature. After the reaction was finished, the catalyst could be readily extracted from the mixture and exhibited effective catalytic activity for a maximum of six cycles.

In recent years, the significance of kinetic studies has grown due to their ability to offer comprehensive insights into reaction pathways and the optimal methods for producing desired products in the chemical industry [25,26].

The motivation for researching the modelling, forecasting, and optimization of transesterification process parameters using RSM is to find the best possible operating conditions for biodiesel synthesis [27]. The RSM method utilises a suitable approximation relationship between input and output variables to identify the optimal conditions for the given process [28,29]. Many researchers have published scientific papers on improving the production of biodiesel by using catalysts that are not in the same phase as the reactants. Taherkani and Sadarmeh [30] conducted an optimization study on the synthesis of linseed biodiesel utilising potassium hydroxide as a catalyst, which led to a biodiesel yield of 93.15 %. The achieved yield was obtained using a catalyst loading of 6.8 wt%, a temperature of 40 °C, a reaction duration of 90 min, and an agitation speed of 700 rpm. Nevertheless, there is a scarcity of information on the modelling and optimization of CD-BaCl-IL catalyst transesterification of linseed oil. However, certain constraints remain, such as the model's incapability to make predictions outside the range of the experiments and deal with intricate variables.

Okeleye and Betiku [31] have reported that soft computing methods, such as ANN and ANFIS, have greater prediction efficiency. The Artificial Neural Network (ANN), modelled like the human brain, possesses the capability to predict complex and nonlinear processes [32] properly. Various studies have employed Artificial Neural Networks (ANN) to simulate biodiesel production processes. Nassef et al. [33] successfully utilised ANFIS modelling to enhance the efficiency of biodiesel production from microalgae. In a similar manner, Ogaga et al. [34] utilised ANFIS modelling to improve the production of biodiesel from Thevetia peruviana seeds. Iweka et al. [35] developed optimal condition for bio oil extraction from ripe paw paw seed as using box-bhenken design and python technique. To the best of our knowledge, no previous investigation has been conducted on the kinetics and soft computing evaluation of LSO transesterification utilising a CD-BaCl-IL catalyst. Therefore, the objective of this study was to evaluate the kinetics and soft computing assessment of LSO transesterification with a CD-BaCl-IL catalyst.

## 2 Materials and method

### 2.1 Materials

Linseed oil was procured at NARICT in Zaria, located at latitude 11°3′N and longitude 7°40′E. Clay was obtained from the Umudike metropolis, 10 km southeast of Umuahia in Abia state, Nigeria, as the precursor material for catalyst preparation due to its accessibility and capacity to form an inert support suitable for impregnation with various functional groups. It is brownish. Barium chloride (Sigma-Aldrich in Poole, England.), necessary for catalyst impregnation, was procured, and Methanol (Merck, Mumbai, India) served as the reactant. 500 ml round bottom flask, glass beads, thermometers, funnels, a three-necked flat bottom flask, burettes (50 ml), conical flasks (250 ml), 500 ml beakers, measuring cylinders, a stopwatch, 1 L separating funnels, a condensation unit, 100 ml storage containers, a hot plate magnetic stirrer, conical flasks (1 L) and a distillation unit.

### 2.2 Characterization of the oil

The ASTM standard [36] was used to characterise the free fatty acid, viscosity, specific gravity, iodine value, acid value, moisture content, peroxide value, ester value, saponification value, and viscosity. FT-IR (model Shimadzu FTIR-8400S) and the GC-MS (model Thermo Finnigan Trace A1300) were employed to identify the functional group and fatty acid profile of the oil, respectively [37].

### 2.3 Alkyl imidazolium ionic liquid synthesis

The synthesis of alkyl imidazolium involves the reaction between alkyl halide and imidazolium salt at a mole ratio of 1:3. The imidazolium salt is initially added to a round-bottom flask, which is then placed in an oil bath heated by a heating mantle. To prevent excessive foaming, the imidazolium salt is progressively mixed with the alkyl halide in the flask. An adapter for a Hoover dryer is connected to the flask in order to eliminate any surplus moisture during the process. The solution is agitated at a rate of 100 rpm and heated to a temperature ranging from 40 to 50 °C for 8 h. Afterwards, the alkyl imidazolium product is gathered and kept at an ambient temperature [30].

### 2.4 Preparation of CD-BaCl-IL catalyst

The clay sample was combined with an ionic liquid and barium chloride at a weight ratio of 2:0.5:0.5. The resulting mixture was subsequently left undisturbed for 12 h. Afterwards, the mixture underwent drying in an oven at a temperature of 105 °C. After the mixture had been dried, it was moved to a porcelain crucible and then covered with a lid. The crucible was subsequently introduced into a muffle furnace, where the mixture underwent carbonisation in the absence of reactive substances at a temperature of 600 °C for 4 h. Ultimately, the final product was placed in a sample holder that was completely sealed to prevent any air or moisture from entering.

### 2.5 Characterization of the raw and modified clay

The physiochemical characteristics of the raw and modified clay were assessed using various analytical techniques. The ASTM D4067 [38] method was employed to evaluate their properties. FT-IR spectroscope was utilised to identify the functional groups present in the samples. XRF analysis was utilised for the elemental composition analysis. XRD was employed to examine the mineralogy of the clay. Lastly, SEM was used to study the morphology of the samples.

### 2.6 Procedure for transesterification

The reaction of, linseed oil, methanol and CD- BaCl-IL resulted in the production of biodiesel, with glycerol being formed as a byproduct. A predetermined amount of oil was meticulously introduced into a flat-bottomed flask positioned on a magnetic stirrer. Next, the exact quantity of methanol was added, coupled with a specific catalyst, determined based on the weight of the oil sample. The flask remained on the magnetic stirrer, ensuring a consistent temperature, while the reaction continued with regulated agitation. At a specified time, the sample was taken out, cooled, and kept undisturbed overnight in normal surroundings, facilitating the separation of the biodiesel (in the upper layer) from the glycerol (in the lower layer). The biodiesel yield was ascertained using the equation illustrated in Equation (1).

1 $$\text{Yield}\;\left(\%\right)=\frac{\text{methylester}\;\text{weight}}{\;\text{oil}\;\text{weight}}\;x\;100$$

The experiment was replicated by adjusting the parameters that affect the transesterification process, including time (1–3 h), catalyst concentration (1–5 wt %), temperature (40–80 °C), agitation speed (150–350 rpm) and methanol/oil molar ratio (4:1–12:1). The process is shown in Fig. 1.

**Fig. 1:** Tranesterification process.

### 2.7 Reaction mechanism for LSO transesterification

The kinetic model employed in this investigation is founded on the LHHW mechanism, which incorporates the surface reaction, adsorption and desorption of molecules and atoms on surfaces [39]. According to Eq. (2), both the reactant molecules T(triglyceride) and A (methanol) are adsorbed at distinct points on the surface of the catalyst. As a result, a chemical reaction takes place between these molecules that are chemically adsorbed, leading to the synthesis of products B (biodiesel) and G (glycerol). Ultimately, the adsorbed products B and G are released from the surface.

(2) $$T+A\;\underset{k_{b}}{\leftarrow }\overset{k_{f}}{\to }\;B+G$$

The transesterification reaction is modelled using the LHHW mechanism, which is presented in Eqs. (3), (4), (5), (6), (7), (8), (9), (10), (11) by Ude and Onukwuli [18]. The mechanism assumption as rate determining step is presented from Eqs. (12), (13), (14), (15), (16), (17), (18), (19), (20), (21), (22) Assumptions for this model include.

i. The catalyst particle size is sufficiently small, so guaranteeing that the reaction is not constrained by diffusion.
ii. The surface's potential for desorption, adsorption or surface reaction is unaffected by coverage, suggesting a homogeneous surface.

(3) $$A+S\;\underset{k_{2}}{\leftarrow }\overset{k_{1}}{\to }\;AS\;\left(Adsorption\;of\;alcohol\right)$$

(4) $$T+S\;\underset{k_{4}}{\leftarrow }\overset{k_{3}}{\to }\;TS\;\left(Adsorption\;of\;triglyceride\right)$$

(5) $$TS+AS\;\underset{k_{6}}{\leftarrow }\overset{k_{5}}{\to }\;DS+BS\;\left(Surface\;reaction\;linking\;triglyceride\;adsorbed\;on\;a\;surface\;with\;alcohol\right)$$

(6) $$DS+AS\;\underset{k_{8}}{\leftarrow }\overset{k_{7}}{\to }\;MS+BS\;\left(Surface\;reaction\;linking\;diglyceride\;adsorbed\;on\;a\;surface\;with\;alcohol\right)$$

(7) $$MS+AS\;\underset{k_{10}}{\leftarrow }\overset{k_{9}}{\to }\;BS+GS\;\left(Surface\;reaction\;with\;monoglyceride\;adsorbed\;on\;a\;surface\;with\;alcohol\right)$$

(8) $$BS\;\underset{k_{12}}{\leftarrow }\overset{k_{11}}{\to }\;B+S\;\left(Desorption\;of\;biodiesel\right)$$

(9) $$DS\;\underset{k_{14}}{\leftarrow }\overset{k_{13}}{\to }\;D+S\;\left(Desorption\;of\;diglyceride\right)$$

(10) $$MS\;\underset{k_{16}}{\leftarrow }\overset{k_{15}}{\to }\;M+S\;\left(Desorption\;of\;monoglyceride\right)$$

(11) $$GS\;\underset{k_{18}}{\leftarrow }\overset{k_{17}}{\to }\;G+S\;\left(glycerol\;desorption\;\right)$$

‘*S’* constitutes the catalyst active site, *D* - diglyceride and M − monoglyceride.

I. Assuming the RDS is alcohol adsorption, Eq. (3)

(12) $$r_{1}=k_{1}\left[A\right]\left[S\right]\;-\;k_{2}\left[AS\right]$$

(13) L=(S)+(TS)+(AS)+(MS)+(DS)+(BS)+(GS)=1

L, which is the Total active site, equals 1

(14) $$r_{1}=\frac{k_{1}\left[A\right]\;-\;\frac{k_{2}\left[D\right]\left[B\right]}{K_{2}K_{3}K_{6}K_{7}\left[T\right]})}{1+\frac{\left[D\right]\left[B\right]}{K_{2}K_{3}K_{6}K_{7}\left[T\right]}+K_{2}\left[T\right]+\frac{\left[D\right]}{K_{7}}+\frac{\left[M\right]}{K_{8}}+\frac{\left[B\right]}{K_{6}}+\frac{\left[G\right]}{K_{9}}}$$

Where $K_{2\;}=\frac{k_{3}}{k_{4}}$, $K_{3\;}=\frac{k_{5}}{k_{6}}$, $K_{4}=\frac{k_{7}}{k_{8}}$, $K_{5\;}=\frac{k_{9}}{k_{10}}$, $K_{6\;}=\frac{k_{11}}{k_{12}}$, $K_{7}=\frac{k_{13}}{k_{14}}$, $K_{8}=\frac{k_{15}}{k_{16}}$,

$$K_{9\;}=\frac{k_{17}}{k_{18}},and\;for\;completeness\;;\;K_{1\;}=\frac{k_{1}}{k_{2}}$$

II. Assuming the RDS is triglyceride adsorption, Eq. (4)

(15) $$r_{2}=\frac{k_{3}\left[T\right]\;-\;\frac{k_{4}\left[D\right]\left[B\right]}{K_{1}K_{3}K_{6}K_{7}\left[A\right]}}{1+K_{1}\left[A\right]+\frac{\left[D\right]\left[B\right]}{K_{1}K_{3}K_{6}K_{7}\left[A\right]}+\frac{\left[D\right]}{K_{7}}+\frac{\left[M\right]}{K_{8}}+\frac{\left[B\right]}{K_{6}}+\frac{\left[G\right]}{K_{9}}}$$

III. Assuming the RDS is the surface reaction linking the adsorbed triglyceride and adsorbed methanol, Eq. (5)

(16) $$r_{3}=\frac{k_{5}{K_{1}K}_{2}\left[T\right]\left[A\right]\;-\;\frac{k_{6}\left[D\right]\left[B\right]}{K_{6}K_{7}}}{{\left(1+K_{1}\left[A\right]+K_{2}\left[T\right]+\frac{\left[D\right]}{K_{7}}+\frac{\left[M\right]}{K_{8}}+\frac{\left[B\right]}{K_{6}}+\frac{\left[G\right]}{K_{9}}\right)}^{2}}$$

IV. Assuming the RDS is the surface reaction linking the adsorbed diglyceride and adsorbed alcohol, Eq. (6)

(17) $$r_{4}=\frac{k_{7}\frac{K_{1}}{K_{7}}\left[D\right]\left[A\right]\;-\;\frac{k_{8}\left[D\right]\left[B\right]}{K_{6}K_{8}}}{{\left(1+K_{1}\left[A\right]+K_{2}\left[T\right]+\frac{\left[D\right]}{K_{7}}+\frac{\left[M\right]}{K_{8}}+\frac{\left[B\right]}{K_{6}}+\frac{\left[G\right]}{K_{9}}\right)}^{2}}$$

V. Assuming the RDS is the surface reaction linking the adsorbed monoglyceride and adsorbed alcohol, Eq. (7)

(18) $$r_{5}=\frac{k_{9}\frac{K_{1}}{K_{8}}\left[M\right]\left[A\right]\;-\;\frac{k_{10}\left[D\right]\left[B\right]}{K_{6}K_{9}}}{{\left(1+K_{1}\left[A\right]+K_{2}\left[T\right]+\frac{\left[D\right]}{K_{7}}+\frac{\left[M\right]}{K_{8}}+\frac{\left[B\right]}{K_{6}}+\frac{\left[G\right]}{K_{9}}\right)}^{2}}$$

VI. Assuming the RDS is biodiesel desorption, Eq. (8)

(19) $$r_{6}=\frac{k_{11}\frac{{K_{1}K_{2}K}_{3}K_{7}\left[T\right]\left[A\right]}{\left[D\right]}\;-\;k_{12}\left[B\right]}{1+K_{1}\left[A\right]+K_{2}\left[T\right]+\frac{{K_{1}K_{2}K}_{3}K_{7}\left[T\right]\left[A\right]}{\left[D\right]}+\frac{\left[D\right]}{K_{7}}+\frac{\left[M\right]}{K_{8}}+\frac{\left[G\right]}{K_{9}}}$$

VII. Assuming the RDS is diglyceride desorption, Eq. (9)

(20) $$r_{7}=\frac{k_{13}\;\frac{{K_{1}K_{2}K}_{3}K_{6}\left[T\right]\left[A\right]}{\left[B\right]}\;-\;k_{14}\left[D\right]\;}{1+K_{1}\left[A\right]+K_{2}\left[T\right]+\frac{\left[B\right]}{K_{6}}+\frac{{K_{1}K_{2}K}_{3}K_{6}\left[T\right]\left[A\right]}{\left[B\right]}+\frac{\left[M\right]}{K_{8}}+\frac{\left[G\right]}{K_{9}}}$$

VIII Assuming the RDS is monoglyceride desorption, Eq. (10)

(21) $$r_{8}=\frac{k_{15}\;\frac{{K_{1}K}_{4}K_{6}\left[D\right]\left[A\right]}{K_{7}\left[B\right]}\;-\;k_{16}\left[M\right]\;}{1+K_{1}\left[A\right]+K_{2}\left[T\right]+\frac{\left[B\right]}{K_{6}}+\frac{{K_{1}K}_{4}K_{6}\left[D\right]\left[A\right]}{K_{7}\left[B\right]}+\frac{\left[D\right]}{K_{7}}+\frac{\left[G\right]}{K_{9}}}$$

IX Assuming the RDS is glycerol desorption, Eq.(11)

(22) $$r_{9}=\frac{\;k_{17}\;\frac{{K_{1}K}_{5}K_{6}\left[M\right]\left[A\right]}{K_{8}\left[B\right]}\;-\;k_{18}\left[G\right]\;}{1+K_{1}\left[A\right]+K_{2}\left[T\right]+\frac{\left[B\right]}{K_{6}}+\frac{\left[D\right]}{K_{7}}+\frac{\left[M\right]}{K_{8}}+\frac{{K_{1}K}_{5}K_{6}\left[M\right]\left[A\right]}{K_{8}\left[B\right]}}$$

Concentrations of D, T, A, M, G and B were evaluated from GCMS analysis utilising equations adopted by Ude and Onukwuli [18] shown in eq. (23)

(23) $$C_{i}\;\left(g/l\right)=5\;X\;10^{-7}\;A+2.1272$$

Where.

$C_{i}$ = concentration of monoglyceride/diglyceride/triglyceride/alcohol/biodiesel/glycerol

A = the peak area of the biodiesel/triglyceride/glycerol/alcohol/monoglyceride/diglyceride evaluated by GCMS.

The rate equations obtained from CD-BaCl-IL were employed as a model for the transesterification process of LSO. The equilibrium and rate constants were evaluated using nonlinear regression equations in the MATLAB environment. The equations were used to find values that minimize the sum of squared differences within the calculated rates and the measured rates for the given data, as shown in Eq. (24). The initial estimates for the rate constant and equilibrium constant were established as 0 and 0.1440, respectively. Polynomial equations were created using GC-MS data to calculate the concentrations of different species participating in the reaction, thereby enabling the determination of each reaction rate. The models were assessed by evaluating their respective variances, which were obtained using Eq. (25), with a 95 % confidence level. The model exhibiting the least variance and having positive parameters exhibited the best fit with the experimental data, whilst the model with the lowest rate constant was determined to be the RDS.

(24) $$S^{2}=\sum {\left(r_{im}-r_{ic}\right)}^{2}$$

(25) $$\sigma^{2}=\frac{S^{2}}{N-K}=\sum_{i=1}^{N}\frac{{\left(r_{im}-\;r_{ic}\right)}^{2}}{N-K}$$

Where $S^{2}$ - the sum of squares, N = no. of runs, K - parameters to be evaluated,

$r_{im}$ - experimental reaction rate for run i, $r_{ic}$ - predicted reaction rate of run i,

$\sigma^{2}$ - variance

The ER model was used to simulate the transesterification kinetics catalyzed by a CD-BaCl-IL. According to this model, the interaction occurs between an adsorbed molecule (T, D, and M in this study) and a non-adsorbed molecule (methanol).

Eley-Rideal steps are developed in seven-step order shown in Eq. (26), (27), (28), (29), (30), (31), (32); the mechanism assumption for the RDS is shown from eq. (33)–(40).

(26) $$T+S\;\underset{k_{2}}{\leftarrow }\overset{k_{1}}{\to }\;TS\;\left(\;triglyceride\;adsorption\right)$$

(27) $$TS+A\;\underset{k_{4}}{\leftarrow }\overset{k_{3}}{\to }\;DS+B\;\left(Surface\;reaction\;linking\;adsorbed\;triglyceride\;and\;alcohol\right)$$

(28) $$DS+A\;\underset{k_{6}}{\leftarrow }\overset{k_{5}}{\to }\;MS+B\;\left(Surface\;reaction\;linking\;adsorbed\;diglyceride\;and\;methanol\;\right)$$

(29) $$MS+A\;\underset{k_{8}}{\leftarrow }\overset{k_{7}}{\to }\;B+GS\;\left(Surface\;reaction\;linking\;adsorbed\;monoglyceride\;and\;methanol\right)$$

(30) $$GS\;\underset{k_{10}}{\leftarrow }\overset{k_{9}}{\to }\;B+S\;\left(glycerol\;desorption\right)$$

(31) $$DS\;\underset{k_{12}}{\leftarrow }\overset{k_{11}}{\to }\;D+S\;\left(\;diglyceride\;desorption\right)$$

(32) $$MS\;\underset{k_{14}}{\leftarrow }\overset{k_{13}}{\to }\;M+S\;\left(\;Monoglyceride\;desorption\right)$$

The ‘*S’* - the catalyst active's site, M − monoglyceride, *D* - diglyceride,

I. Assuming the RDS is triglyceride adsorption, Eq. (26)

L = (S) + (TS) + (AS) + (MS) + (DS) + (BS) + (GS) = 1 (33)

L, which is the Total active site, equals 1

(34) $$r_{1}=\frac{k_{1}\left[A\right]\;-\;\frac{k_{2}\left[D\right]\left[B\right]}{K_{2}K_{6}\left[A\right]}}{1+\frac{\left[D\right]\left[B\right]}{K_{2}K_{6}\left[A\right]}+\frac{\left[G\right]}{K_{5}}+\frac{\left[D\right]}{K_{6}}+\frac{\left[M\right]}{K_{7}}\;}$$

II. Assuming the RDS is a surface reaction linking adsorbed triglyceride and non-adsorbed alcohol, Eq. (27)

(35) $$r_{2}=\frac{k_{3}K_{1}\left[T\right]\left[A\right]\;-\;\frac{k_{4}\left[D\right]\left[B\right]}{K_{6}}}{1+K_{1}\left[T\right]+\frac{\left[G\right]}{K_{5}}+\frac{\left[D\right]}{K_{6}}+\frac{\left[M\right]}{K_{7}}}$$

III. Assuming the RDS is a surface reaction linking adsorbed diglyceride and non-adsorbed alcohol, Eq. (28)

(36) $$r_{3}=\frac{k_{5}\frac{\left[D\right]\left[A\right]}{K_{6}}]\;-\;\frac{k_{6}\left[M\right]\left[B\right]}{K_{7}}}{1+K_{1}\left[T\right]+\frac{\left[G\right]}{K_{5}}+\frac{\left[D\right]}{K_{6}}+\frac{\left[M\right]}{K_{7}}}$$

IV. Assuming the RDS is a surface reaction linking adsorbed monoglyceride and non-adsorbed alcohol, Eq. (29)

(37) $$r_{4}=\frac{k_{7}\frac{\left[M\right]\left[A\right]}{K_{7}}\;-\;\frac{k_{8}\left[G\right]\left[B\right]}{K_{5}}}{1+K_{1}\left[T\right]+\frac{\left[G\right]}{K_{5}}+\frac{\left[D\right]}{K_{6}}+\frac{\left[M\right]}{K_{7}}}$$

V. Assuming the RDS is glycerol desorption, Eq. (30)

(38) $$r_{5}=\frac{\;k_{9}\frac{K_{4}\left[M\right]\left[A\right]}{K_{7}\left[B\right]}\;-\;k_{10}\left[G\right]}{1+K_{1}\left[T\right]+\frac{\left[D\right]}{K_{6}}+\frac{\left[M\right]}{K_{7}}+\frac{K_{4}\left[M\right]\left[A\right]}{K_{7}\left[B\right]}}$$

VI. Assuming the RDS is diglyceride desportion, Eq. (31)

(39) $$r_{6}=\frac{k_{11}\;\frac{K_{1}K_{2}\left[T\right]\left[A\right]}{\left[B\right]}\;-\;k_{12}\left[D\right]\;}{1+K_{1}\left[T\right]+\frac{K_{1}K_{2}\left[T\right]\left[A\right]}{\left[B\right]}+\frac{\left[M\right]}{K_{7}}+\frac{\left[G\right]}{K_{5}}}$$

VII. Assuming the RDS is monoglyceride desorption, Eq. (32)

(40) $$r_{7}=\frac{k_{13}\;\frac{K_{8}\left[D\right]\left[A\right]}{K_{6}\left[B\right]}\;-\;k_{14}\left[M\right]\;}{1+K_{1}\left[T\right]+\frac{K_{8}\left[D\right]\left[A\right]}{K_{6}\left[B\right]}+\frac{\left[D\right]}{K_{6}}+\frac{\left[G\right]}{K_{5}}}$$

### 2.8 Determination of thermodynamic properties

The Activation energy for the RDS was determined using the Arrhenius eq. in Eq. (41).

(41) $$k=A\;e^{\frac{-E_{a}}{RT}}$$

Eq. (41) linearization gave Eq. (42). slope - *Ea/R* and intercept - *lnA.* were determined plot of ln *k* against *(1/T)*

(42) $$lnk=\left(\;\frac{-E_{a}}{RT}\;\right)+lnA$$

Ea - activation energy (J/mol), *k* - rate constant, R -gas constant (8.314 Jmol/K), *A* - pre-exponential factor, T - temperature (K).

The study aimed to assess the impact of five specific variables, including the methanol/oil mole ratio, catalyst dosage, temperature, time, and agitation speed, on the formation of biodiesel. Table 1 presents the experimental design and levels of the independent variables. The selected dependent variable was the yield of biodiesel. To ensure precise error estimations, eight replications of the centre points were carried out, and the experiments were completed in a randomised sequence.

**Table 1:** Overview of the design considerations for the transesterification process.

Factor	Units	Low level	Mid-low level	Mid-level	Mid-high level	High level
Catalyst dosage, (A)	wt%	1(-2)	2(-1)	3(0)	4(+1)	5(+2)
Methanol/oil ratio, (B)	mol/mol	4:1(-2)	6:1(-1)	8:1(0)	10:1(+1)	12:1(+2)
Time, (C)	hour	1(-2)	1.5(-1)	2(0)	2.5(+1)	3(+2)
Temperature, (D)	^o^C	40(-2)	50(-1)	60(0)	70(+1)	80(+2)
Agitation speed, (E)	rpm	150(-2)	200(-1)	250(0)	300(+1)	350(+2)

### 2.9 ANN model development

ANN model was developed to execute tasks that mimic the functions of the brain using biological neurons. Testing, validation, and model training were essential elements of this undertaking. The idea of backpropagation was employed to elucidate the feed-forward mechanism in a multilayer perceptron. The network is composed of five layers: an output layer containing the biodiesel yield (%), an input layer containing the catalyst dose (wt%), time (hour), methanol/oil ratio (mol/mol), temperature (^o^C), and agitation speed (rpm), and a hidden layer consisting of ten neurons. The collected data was divided into three distinct groups, allocated with proportions of 70 %, 15 %, and 15 %, respectively. These groups were utilised for training the network, validating the results, and testing the network, as stated in Ref. [40]. Fig. 2 illustrates the structure of the ANN.

**Fig. 2:** ANN basic structure.

### 2.10 ANFIS modelling

A fuzzy model [41] was used to forecast the transesterification process. This study utilised a single output (biodiesel yield) and five independent factors: catalyst dosage (expressed as a weight percentage), methanol/oil ratio (measured in moles per mole), time (measured in hours), temperature (measured in degrees Celsius), and agitation speed (measured in revolutions per minute). The purpose was to model non-linear variables. The modelling process utilised MATLAB R2015b′s fuzzy logic toolbox. Fig. 3 depicts the design of the five-level Adaptive Neuro-Fuzzy Inference System (ANFIS) as presented in Ref. [38].

**Fig. 3:** ANFIS basic structure.

### 2.11 Developed model's evaluation

The model's evaluation for the process was assessed using the parameters presented below in equations (43), (44)).

(43) $$MSE=\frac{1}{P}\sum_{p=1}^{p}{\left(d_{p}-O_{p}\right)}^{2}$$

(44) $$R^{2}=1-\frac{\sum_{p=1}^{p}{\left(d_{p}-O_{p}\right)}^{2}\;}{\sum_{p=1}^{p}{\left(O_{p}\right)}^{2}\;}$$

$d_{p}$ and o_p_ denote the experimental and predicted values. The proximity of the MSE value to zero and the R^2^ value to one indicates the high efficiency of the models [42].

## 3 Results and discussion

### 3.1 Physicochemical properties of linseed oil

Table 2 presents the physiochemical properties of raw linseed oil. The oil has acid values of 8.98mgKOH/g and 4.49 % for free fatty acid. These results exhibit a relatively high level in the context of one-step transesterification, which requires pre-treatment of the oil to reduce soap generation and enhance glycerol separation. The saponification and peroxide values of the oil are indicators of its ability to withstand rancidity. The iodine value of 81.6gI_2_/100 g indicates the existence of unsaturated triglycerides in the oil.

**Table 2:** Characteristics of oils related to their physicochemical properties.

Physicochemical properties	Linseed oil
Oxidation stability 110°C (Hour)	4.2
Peroxide value	4.78
Free fatty acid (FFA) (%)	4.449
Flash point	59
Iodine value (gI_2_/100 g)	81.6
Saponification value (mgKOH/g)	253.49
Kinematic viscosity at 40°C (mm^2^/s)	57.34
Cloud point	−2.89
Moisture content (%)	0.17
Pour point	−3.17
Specific gravity	0.88
Refractive index	1.46
Acid value (mg/OH)	8.98
Molecular weight	688.30

Nevertheless, the elevated viscosities and densities of both oils render them inappropriate for direct utilisation as biofuels, as they obstruct the process of atomization in internal combustion engines [43]. The oxidation stability of linseed oil is determined to be high and falls below the ASTM D6751 requirement (3 h), potentially as a result of the extraction technique utilised [44]. The kinematic viscosity of linseed oil, which is 57.34, is similar to the value reported by Tariq et al. [45] (30.43) and 31.61 by Balamurugan et al. [46] on linseed oil characterization. This indicates that linseed oil has favourable fuel quality and shows promise as a feedstock. The substance has a high viscosity and may have a sluggish rate of flow.

### 3.2 FT-IR of linseed oil

The FTIR spectrum of linseed oil, as depicted in Fig. 4, was analysed to determine the different functional groups present in the raw material. The presence of = C-H functional groups (alkenes) is indicated by the peak observed at 749.2 cm^−1^ in the spectrum. The spectrum's low energy and frequency range strongly indicate the presence of double-bonded bending vibrations in these functional groups [47]. The vibrations are a result of unsaturated olefinic (alkene) functional groups, which are present in unsaturated fatty acid methyl esters found in biodiesel, such as methyl oleate and methyl linoleate [4]. Furthermore, the appearance of clearly defined peaks at 995.2 cm^−1^ indicates the existence of stretching vibrations in the C-O and C-O-C molecules. Furthermore, the spectrum [48] can also reveal the bending vibration of O-CH_3_. The band detected at 1114.5 cm^−1^ corresponds to the bending vibrations of C=C bonds, while the band at 1025.0 cm^−1^ is attributed to the bending vibrations of C-H methyl groups [40]. The peak suggests the presence of a blend of aromatic compounds at 1640.0 cm^−1^. The identification of an O-H group in carboxylic acid is indicated by the signal at 2776.9 cm^−1^ in the spectra. The peaks detected at 2881.2 cm^−1^ are attributed to the symmetric stretching vibrations of the C-H alkane groups. Unlike the typical low-energy and frequency ranges where the C-H bending vibrations of alkene groups are observed, certain groups like methyl (CH_3_) or methylene groups require a significant amount of energy to induce stretching vibrations within their bond [49]. The peak observed at 3652.8 cm^−1^ is ascribed to the stretching vibration of alkene groups with = C-H bonds.

**Fig. 4:** Linseed oil FT-IR analysis.

### 3.3 Linseed oil's fatty acid constituent

The fatty acid profile of linseed oil was analysed using GC-MS. Table 3 displays the fatty acid content of linseed oil, indicating that it consists of 86.5 % unsaturated acids and 13.547 % saturated acids. According to Qasemi et al. [50], the oil is classified as oleic acid because it mostly contains linolenic acid, which makes up 56.5 % of the total fatty acid content, and linoleic acid, which makes up 14 %. This indicates that the oil contains a significant quantity of unsaturated fatty triglycerides that are appropriate for transesterification [51]. Additionally, it was noted that the fatty acid makeup of the oil closely approximated that of conventional oils commonly utilised in the synthesis of biodiesel [52].

**Table 3:** Linseed oil's fatty acid composition.

S/N	FFA Profile		Linseed oil
	Fatty Acid	Component	Composition (%)
1	Capric acid	C_10_	–
2	Lauric acid	C_12_	0.25
3	Myristic acid	C_14_	3.51
4	Palmitic acid	C_16:0_	5.91
5	Stearic acid	C_18:0_	3.31
6	Oleic acid	C_18:1_	16
7	Linoleic acid	C_18:2_	14
8	Linolenic acid	C_18:3_	56.5
9	Arachidic acid	C_20_	0.567
	Total		100.047

### 3.4 Analysis of the synthesized catalyst's characteristics

#### 3.4.1 Synthesized catalyst's physiochemical properties

Table 4 displays the physical characteristics of both the unaltered and altered clay catalysts. The clay's characteristics were enhanced after being activated with BaCl and an ionic liquid. Consequently, there was a rise in the extent of the exposed surface, facilitating the more effortless spread of reactants throughout the inner regions of the catalyst. Furthermore, a greater pore volume of 24.23 was achieved. The pore size of the raw clay also enlarged following various forms of activation. The increase in pore size can be attributed to either an increase in the porosity of the synthesized material or the formation of secondary pores resulting from the interaction between BaCl, the ionic liquid, or the clay [38,50].

**Table 4:** Synthesized clay catalyst's physical properties.

Parameters	Raw Clay	CD-BaCl-IL
Surface area (m^2^/g)	284.286	363.297
Pore size (nm)	2.680	3.140
Total pore volume (cm^3^/g)	24.11	24.23

#### 3.4.2 FTIR analysis of the synthesized catalyst

The FTIR spectroscope was employed to analyse the functional groups present in the unprocessed clay catalyst, CD-BaCl-IL. The results are illustrated in Fig. 5, Fig. 6. Upon examination of the figure and table, it is evident that both catalysts exhibit comparable functional groups, including Si-O-Si, C-Cl of aliphatic chloro compounds, C-H stretch of aromatic bend, C-H stretch of vinyl, organic silicone Si-O-C, Si-O, double bond C=C at a wavenumber of.

**Fig. 5:** FTIR evaluation of raw clay.

**Fig. 6:** FTIR evaluation of CD-BaCl-IL.

2855 cm^−1^, and -OH stretch of primary alcohol at a wavenumber of 3004 cm^−1^, and Al–OH–Al vibrations [40]. When comparing the raw clay and CD-BaCl-IL, it is clear that there is no significant reduction in the intensity of the bands at 693.3 cm^−1^ for raw clay and at 723.1 cm^−1^ for CD-BaCl-IL. This implies that the alterations performed have resulted in relatively minor adjustments to the structure. The FTIR bands observed at a wavenumber of 913.2 cm^−1^ are indicative of the existence of Al–O.H.–Al in the unprocessed Clay [51]. The modification process led to a decrease in the intensity of these bands due to the leaching of octahedral cations (Al^3+^) from the clay structure [47]. The occurrence of unbound silica in both untreated clay and CD-BaCl-IL catalysts is linked to the bending of Si-O-Si bonds at wave numbers of 693.3 cm^−1^ and 723.1 cm^−1^, respectively. In addition, the stretching of Si-O in the plane is observed at wave numbers of 1032.5 cm^−1^ for raw Clay and 1166.7 cm^−1^ for CD-BaCl-IL catalysts. The raw clay catalyst contains cyanide ions that can hinder the catalytic activity of the clay. Nevertheless, the inclusion of BaCl and an ionic liquid in the clay eradicates the existence of cyanide [53].

#### 3.4.3 Synthesized catalysts using SEM

The morphologies of the raw clay catalyst and CD-BaCl-IL are depicted in Fig. 7, Fig. 8, respectively. The micrographs of the CD-BaCl-IL revealed an augmentation in both the quantity and size of pores on the Clay. Their physical structure exhibited greater clumping together; the presence of additional openings on the clay particles was detected in CD-BaCl-IL, which indicates that it possesses a larger surface area with smaller pore dimensions; the scanning electron microscope (SEM) findings align with the results reported by Ude and Onukwuli [54] In relation to an alkaline activated clay catalyst development for the transesterification of gmelina oil.

**Fig. 7:** SEM of unprocessed clay.

**Fig. 8:** SEM of clay impregnated with BaCl-ionic liquid.

#### 3.4.4 XRF analysis

The chemical composition of the raw Clay and CD-BaCl-IL used in this study is specified in Table 5. The main components of Clay consist of silicon (Si), aluminium (Al), titanium (Ti), and iron (Fe). The substance consists of metallic oxides, specifically Al_2_O_3_, SiO_2_, TiO_2_, Cr_2_O_3_, Mn_2_O_3_, Fe_2_O_3_, and ZnO. The oxides mentioned are crucial constituents of heterogeneous catalysts [54,55]. The clay included a significant amount of SiO_2_, and the introduction of CD-BaCl-IL led to a notable rise in the concentrations of BaO and Cl due to the modification. The incorporation of BaCl and ionic liquid into the untreated Clay led to a decrease in the quantity of SiO_2_. The reduction in the amount of Al_2_O_3_ led to the categorization of the altered Clay as Brønsted and Lewis acids. The acidity and catalytic abilities of the clay are mostly dependent on the electronegativity of the interlamellar spacing of exchangeable cations that are linked to the negatively charged aluminosilicate sheets. Consequently, the activation process led to an increase in both the number and strength of Brønsted and Lewis acid sites [56,57].

**Table 5:** XRF of the synthesized catalysts.

Elements	RC	CD-BaCl-IL
SiO_2_	62.051	58.503
V_2_O_5_	0.189	0.249
Cr_2_O_3_	0.056	0.052
MnO	0.035	0.031
Fe_2_O_3_	3.971	4.113
CO_3_0_4_	0.018	0.021
NiO	0.004	0.003
CuO	0.042	0.045
Nb_2_O_3_	0.034	0.041
SO_3_	0.341	0.171
CaO	0.331	0.256
K_2_O	0.228	0.222
BaO	0.130	3.676
Al_2_O_3_	27.323	26.485
Ta_2_O_5_	0.030	0.046
TiO_2_	4.354	4.294
ZnO	0.009	0.010
Ag_2_O	0.027	0.018
Cl	0.561	1.497
ZrO_2_	0.265	0.266

#### 3.4.5 XRD analysis

Fig. 9, Fig. 10 show the X-ray diffraction patterns of the clay in its original form and the CD-BaCl-IL catalyst. The diffractogram reveals a clear peak at approximately 2θ = 27° for clay, 27.5°, and 28.1° for CD-BaCl-IL. These slight changes indicate that the untreated clay was effectively modified with BaCl and ionic solutions. Fig. 8 confirms that the clay belongs to the kaolinite group, providing evidence of the presence of alumina and silica. Additionally, the presence of quartz in the clay suggests that it is a residual clay originating from its source. The addition of CD-BaCl-IL results in the formation of garnet, which can be attributed to the presence of BaCl and the ionic liquid used in the modification process [[58], [59], [60]].

**Fig. 9:** XRD analysis of the raw Clay.

**Fig. 10:** XRD analysis of the CD-BaCl-IL.

### 3.5 Process parameters impacts

#### 3.5.1 Effect of catalyst dosage

Catalysts offer alternate routes for the cleavage of chemical bonds. Fig. 11 illustrates the impact of catalyst dosages, measured as the weight % of the LSO, on the yield. The yield of methyl ester rose as the catalyst weight rose, reaching a peak at four wt%. Beyond this point, the yield began to reduce. This can be explained by the fact that a catalyst dosage of 4 wt% provides the highest number of active sites for the interaction of reactants, leading to a significant increase in the rate of mass transfer within the three-phase system (alcohol, oil, and catalyst). The enhanced productivity of the methyl ester resulting from an augmented catalyst weight can be attributed to the heightened availability of the catalyst inside the reaction medium. Nevertheless, there was no additional enhancement observed in the production of biodiesel when the amount of catalyst used exceeded 4 wt%. The potential cause could be an elevation in the viscosity of the multiphase system, impeding their proper blending. This observation is consistent with the report of Alaba et al. [61] about the manufacture of methyl ester from shea butter.

**Fig. 11:** Effect of catalyst dosage on LSO biodiesel yield.

#### 3.5.2 Methanol/oil ratio effect

The stoichiometric ratio of methanol to oil is a crucial factor that greatly influences the production efficiency of methyl esters. The stoichiometry of the transesterification process normally requires a molar ratio of 3:1 between methyl ester and glycerol. Nevertheless, a significant quantity of alcohol is required to facilitate the reaction. The effect of the molar ratio, varying from 4:1 to 12:1, on the clay catalyst was investigated while keeping the other process parameters consistent in Fig. 12. The results indicated that the methanol/oil molar ratio significantly affects the synthesis of methyl ester. The optimal ester yield was obtained by employing a methanol/oil molar ratio of 10:1; the raw clay catalyst had the lowest yield. An elevated molar ratio resulted in a higher yield of biodiesel. The increased methanol concentration led to a substantial increase in the yield, causing the reaction to produce the desired product preferentially. The yield declined when the molar ratio surpassed 10:1, potentially due to the reconversion of the fatty acid methyl ester into triglycerides. Another potential factor is the presence of methanol, which contains a polar hydroxyl group that functions as an emulsifier. This emulsification process makes it difficult to separate the ester layer from the water layer, particularly when a significant amount of methanol is used. As a result, the ester's yield decreased [61,62].

**Fig. 12:** Methanol/oil ratio effect on LSO methyl ester yield.

#### 3.5.3 Effect of time

The biodiesel's % yield exhibited a positive correlation with the duration of the reaction. This study examined the impact of the duration between 0 h and 3 h on the production of LSO biodiesel, as shown in Fig. 13, specifically focusing on the biodiesel yield. The study revealed that the optimal reaction time for the LSO biodiesel was 2 h, resulting in a higher yield. However, any reaction time above 2 h led to a reduction in the yield. The reaction exhibited a significant deceleration as a result of the methanol and triglycerides diffusion into catalyst active sites. The observed reduction in yield after 2 h may be attributed to a reversible transesterification reaction, leading to the depletion of esters [30,36].

**Fig. 13:** Effect of time on the output of LSO biodiesel.

#### 3.5.4 Temperature effect on the methyl ester yield

Fig. 14 investigates the impact of temperature on the production of methyl ester during the transesterification process of LSO biodiesel using CD-BaCl-IL. The temperature was varied between 40 °C, 50 °C, 60 °C, 70 °C, and 80 °C, while keeping all other parameters constant. The reaction rate decreased at lower temperatures, but the highest yield of methyl ester was observed at 60 °C. This suggests that increasing the reaction temperature reduces the oil's viscosity, improves mass transfer between phases, and enhances the frequency and strength of collisions between reactant molecules. The decrease in yield can be attributed to the evaporation of methanol at higher temperatures during the reaction [[61], [62], [63]]. This finding aligns with Ajala et al.'s [64] study on LSO biodiesel optimization.

**Fig. 14:** Temperature effect on LSO methyl ester yield.

#### 3.5.5 Effect of agitation speed

Mixing guarantees uniformity throughout the reaction mixture. The study conducted by Dadhnaia et al. [24] found that it enhanced the surface area of contact between oils and catalyst or methanol solution. Mixing additionally enhances the response. Fig. 15 displays the yield of methyl esters obtained from LSO biodiesel using CD-BaCl-IL at various agitation rates. The data indicates that the highest biodiesel output was achieved when the agitation speed was set at 300 rpm for all catalysts and the biodiesel. It is possible that increasing the mixing intensity favoured the occurrence of the backward reaction [25]. The CD-BaCl-IL catalyst outperformed the raw clay due to the introduction of dopants, which enhanced its surface area and porosity. The raw clay catalysts exhibited the lowest performance, indicating the necessity to enhance their catalytic activity through activation and doping.

**Fig. 15:** Effect of agitation speed on LSO biodiesel yield.

### 3.6 Distribution of the products

Fig. 16 (a, b, and c) shows the changes that occur in the reactants that are being transformed into products during the process of transesterification of LSO using CD-BaCl-IL catalyst at temperatures of 40°C, 50°C, and 60. The reaction was performed with the following parameters: a methanol/oil molar ratio of 10:1, a catalyst dosage of 4 wt%, a time of 2 h, and an agitation speed of 300 rpm. The transesterification reaction occurred via a sequence of consecutive, reversible reactions. The data unequivocally illustrates that the levels of biodiesel and glycerol increased over time while the levels of the reactants (monoglyceride, diglyceride, triglyceride, and alcohol) decreased during the same period. Substantial variations in the concentration of both products and reactants were observed at all temperatures. The data also shows that methyl ester is the prevailing component in the product, especially at a temperature of 60°C. The results suggest that a greater yield is obtained when the temperature is set at 60 C. The heightened concentration of unsaturated free fatty acids can elucidate the occurrence. In addition, the inclusion of a co-solvent aids in the creation of a phase that is rich in glycerol during the reaction. During this phase, the catalyst is able to migrate into the glycerol phase, causing a decrease in the concentration of the catalyst in the ester phase. As a result, the decrease in catalyst concentration decelerates the reaction rate [39,64,65].

**Fig. 16:** Species concentration against time for LSO transesterification catalyzed by CD-BaCl-IL for a. 40°C, b. 50°C and c. 60°C.

### 3.7 Kinetics study

The results of the study on the transesterification process of LSO using a heterogeneous (CD-BaCl-IL) catalyst have been recorded in Table 7, Table 8. The evaluation employed two non-elementary reaction mechanisms: LHHW and ER. For the LHHW process, we investigated nine different kinetic models that considered the adsorption, surface reaction, and desorption of species. In addition, seven models were used to evaluate ER. The equilibrium and rate constants were determined using nonlinear regression analysis with MATLAB 2014 software. The goal was to determine the optimal values of these parameters that minimize the sum of squared disparities between the measured rates and the calculated rates for the given data. The initial values for the constants were set at 0.0370 and 0.1440, as reported by Ajala et al. [64]. The model equation was utilised to ascertain the reaction rate for each species, and their concentrations were acquired using GC-MS analysis. The model was evaluated by comparing it using statistical indicators, specifically variance. The RDS is characterised by having the lowest variance in kinetic and equilibrium constants, as well as exhibiting more positive parameters. The equilibrium and rate constants derived at different temperatures are presented in Table 7 for the LHHW model and Table 8 for the ER model. The LHHW model exhibited the lowest value of variance (2.61E-14) at 40°C in the surface reaction connecting adsorbed triglyceride and adsorbed alcohol as the RDS, leading to the most accurate alignment with the experimental results. Conversely, the ER model exhibited the least amount of variance (3.78E-12) at 60°C in the surface reaction between alcohol that is not adsorbed and triglyceride that is adsorbed, leading to the most accurate fit. Thus, these reactions might be regarded as the RDS. This supports the theory that more than 75 % of all heterogeneous reaction mechanisms are predominantly controlled by surface reactions [1]. Table 6, Table 7 presented the thermodynamic properties of the RDS. It was observed that the rate constant showed a positive correlation with temperature, suggesting that the reaction is endothermic. The references cited are derived from the publications of diBitonto et al. [66] and Ude et al. [18], and Zhao et al. [1]. Empirical observations suggest that the LHHW model offers a more precise depiction of the kinetic data in comparison to the ER model. This is corroborated by an R^2^ of 0.9999 compared to 0.9475 for the ER model, indicating a strong relationship between the variables as seen in Table 8. Hence, the model demonstrates a good fit, This finding aligns with the investigation carried out by Onukwuli and Ude [18] on the kinetic evaluation of the transesterification process of gmelina seed oil.

**Table 6:** Rate constants with thermodynamics data for LSO biodiesel via the LHHW model.

	40^O^C	50^O^C	60^O^C	△E (kJ/mol)	A
k_5_(hr^−1^)	0.1287	0.1381	0.1629	10.22	6.41
k_6_(hr^−1^)	2.762	2.876	4.391	19.97	5.5E3
K_1_	0.061	0.134	0.250	61.79	1.22E9
K_2_	0.0674	0.1144	0.5431	90.43	6.61E13
K_6_	0.0447	0.3819	1.2988	147.997	2.31E23
K_7_	0.1748	1.0452	1.323	89.67	1.93E14
K_8_	0.152	0.112	0.211	13.61	7.17E13
K_9_	0.85	0.819	0.314	42.82	1.3E7
Variance	5.73E-9	2.61E-8	4.47E-9

**Table 7:** Rate constants with thermodynamics data for LSO biodiesel via ER model.

	40^O^C	50^O^C	60^O^C	△E, △H (kJ/mol)	A, △S (J/molk)
**k**_**3**_**(hr**^**−**^**^1^)**	0.1754	0.1913	0.5674	50.5	3.9E7
**k**_**4**_**(hr**^**−**^**^1^)**	0.1343	0.1439	0.1739	11.20	9.68
**K**_**1**_	0.1071	0.1172	−0.1530	15.45	3.9E1
**K**_**2**_	−0.0602	0.0625	0.0690	41.08	4.4E6
**K**_**6**_	0.0894	0.0748	0.0620	15.98	5.1E3
**K**_**7**_	0.0214	−0.0720	0.0818	58.62	1.52E8
**Variance**	2.38E-11	2.38E-10	2.02E-9

**Table 8:** Comparison of the parameters for the LHHW and ER model.

Reaction mechanism	Temperature	Variance	R^2^
LSO catalyzed by CD-BaCl-IL ER model	40^O^C	2.38E-11	0.7805
	50^O^C	2.38E-10	
	60^O^C	2.02E-9	
LSO catalyzed by CD-BaCl-IL LHHW model	40^O^C	5.73E-9	0.9348
	50^O^C	2.61E-8	
	60^O^C	4.47E-9	

### 3.8 Modelling and simulation

The computed equilibrium and rate constants were used in the rate-determining step (RDS) equation (16)(r3) for LHHW to forecast the reaction rate in terms of the conversion of triglyceride. This prediction was then simulated using MATLAB version 2014 and represented graphically in Fig. 17. The figure indicates a strong correlation linking the experimental and predicted values. Therefore, the rate expression in terms of conversion based on the surface reaction linking triglyceride and adsorbed alcohol, which is the RDS in the LHHW elementary mechanism, is the most statistically accurate depiction of the empirical data for transesterification. This phenomenon may be attributed to the fact that triglycerides are relatively large molecules and possess lower polarity compared to methanol, resulting in their slow adsorption. Consequently, this delayed adsorption becomes the limiting factor in the process [18].

**Fig. 17:** Triglyceride conversion prediction against time LSO biodiesel synthesis for LHHW (RDS) at different temperatures.

### 3.9 Modelling via RSM, ANN and ANFIS

Yield of LSO FAME by CD-BaCl-IL = 80.0477–2.03833A + 0.285B + 0.6075C −1.0075D + 2.71167E + 1.42 AB + 1.53875 AC -0.6475AD −1.94AE −0.19125 BC + 0.35BD + 0.05 BE + 2.15625 CD -0.58625CE + 1.4175 DE + 0.211023 A^2^ + 0.211023 B^2^ + 0.211023C^2^ + 0.211023 D^2^ + 0.211023 E^2^ (45)

Table 9 presents a matrix of the operational parameters that affect the production of linseed oil. The results show that these variables significantly influence the outcome. To establish a relationship between the parameters of the linseed biodiesel process and generate the model equations mentioned earlier, a quadratic polynomial was used to fit the provided data. Biodiesel production is influenced by several independent factors, including catalyst concentration (A), methanol/oil molar ratio (B), reaction temperature (C), reaction time (D), and agitation speed (E). The parameters for the transesterification reaction were predicted using Response Surface Methodology (RSM). A total of thirty-two experimental conditions were created using the Central Composite Design (CCD) to determine how each variable affects the response. The coefficient of the quadratic polynomial regression model for the response, as shown in equation (45), was determined using various regression approaches. The one-factor coefficient indicates the impact of each specific variable, while the interaction between two variables and the quadratic influence is represented by the two-factor and second-order coefficients [28,67]. The congruity between the observed and anticipated outcomes (RSM, ANN, and ANFIS) confirmed the adequacy of the model. The models' ability to forecast the process was demonstrated [68,67].

**Table 9:** Experimental run for CD-BaCl-IL transesterification process of LSO.

Run	A: catalyst con. Wt. %	B: methanol/oil ratio mol/mol	C: time hour	D: temperature ^o^C	E: agitation speed rpm	biodiesel yield %	RSM predicted (biodiesel yield)	ANN predicted yield	ANFIS predicted yield
1	2	6	2.5	70	400	91.2	90.05	90.05	90.0493
2	4	6	2.5	50	400	78.55	77.55	77.67	77.54972
3	3	8	2	60	500	86.11	86.11	86.11	86.11016
4	3	4	2	60	300	80.07	80.07	80.12	80
5	3	8	3	60	300	82.34	82.34	82.36	82.3399
6	4	6	2.5	70	200	78.59	78.59	78.59	78.58924
7	4	10	1.5	70	200	72.87	72.87	72.86	72.86998
8	2	10	2.5	70	200	77.91	77.91	77.96	77.90953
9	2	6	1.5	50	400	92.1	89.78	89.78	89.77918
10	1	8	2	60	300	84.88	84.88	85.04	84.88014
11	3	8	2	60	300	80	80	80.02	80.00007
12	3	8	2	60	300	80	80	80.02	80.00007
13	4	10	2.5	70	400	85.46	85.46	85.45	85.45925
14	2	10	1.5	50	200	81.49	81.49	81.62	81.48942
15	3	8	2	60	300	80	80	80.01	80.00007
16	4	10	1.5	50	400	81.92	81.92	81.91	81.91949
17	2	6	2.5	50	200	79.52	79.52	79.51	79
18	3	8	2	60	300	80	80	80.02	80.00007
19	3	8	2	40	300	82.44	82.44	82.46	82.44015
20	5	8	2	60	300	77.19	77.19	77.2	77.19012
21	2	10	2.5	50	400	81.44	81.44	81.6	81.43987
22	2	10	1.5	70	400	88.1	88.1	88.1	88.09947
23	4	6	1.5	50	200	79.25	79.25	79.3	79.24957
24	4	6	1.5	70	400	74.3	74.3	74.29	74.29998
25	3	12	2	60	300	82	82	81.99	82.00015
26	3	8	2	60	300	80	80	80.02	80.00007
27	3	8	2	60	300	80	80	80.02	80.00007
28	3	8	1	60	300	79.73	79.73	79.69	79.72991
29	4	10	2.5	50	200	82.97	82.97	82.83	82.96943
30	3	8	2	80	300	79.63	79.63	79.6	79.63014
31	3	8	2	60	100	75.96	75.96	76.01	75.96014
32	2	6	1.5	70	200	76	76	76.02	75.99981

The analysis of variance results is presented in Table 10. The model's R^2^, adjusted R^2^, and predicted R^2^ values were 0.9947, 0.9850, and 0.8594, respectively. These values indicate a strong fit for the model and a positive correlation between the observed and predicted values. The overall model showed statistical significance with a p-value of less than 0.05. The single, interaction, and quadratic terms were found to be significant, except for BC, BE, C^2^, and E^2^, which were deemed unimportant. These findings suggest that all of the process factors had a significant impact on the transesterification of linseed oil. The model's standard deviation of 0.5286, mean of 81.10, coefficient of variation (C.V%) of 0.6518 %, less than 10 %, and accuracy of 44.6 indicate that the model is acceptable and robust for optimization. The cor. total of 577.76 which refers to the amount of variation around the mean, aligns with the overall model (574.69), showing a good fit for the model; a pure error of 0 indicates there is no variability within the process, PRESS (81.25), which refers to the predicted residual error sum of squares aligns with the mean (81.10) with a slight variation showing a good fit for the model. The lack of fit for the model, with a value of 0.5123, was found to be statistically insignificant, further validating the appropriateness of the model. These results are consistent with previous research conducted by Olatunji et al. [29] on the conversion of shea butter oil into biodiesel through transesterification, Ajala et al. [64] on the enhancement of two stages of biodiesel synthesis from shea butter oil, and Roberto Cardoso Bastos et al. [69] on the use of sulfonated catalyst derived from agricultural waste for biodiesel production.

**Table 10:** ANOVA model of linseed biodiesel via CD-BaCl-IL.

Source		Sum of Squares	df	Mean Square	F-value	p-value	
Model		574.69	20	28.73	102.83	<0.0001	significant
A		99.72	1	99.72	356.85	<0.0001	
B		1.95	1	1.95	6.98	0.0229	
C		8.86	1	8.86	31.70	0.0002	
D		24.36	1	24.36	87.18	<0.0001	
E		176.48	1	176.48	631.55	<0.0001	
AB		32.26	1	32.26	115.46	<0.0001	
AC		37.88	1	37.88	135.58	<0.0001	
AD		6.71	1	6.71	24.01	0.0005	
AE		60.22	1	60.22	215.50	<0.0001	
BC		0.5852	1	0.5852	2.09	0.1757	
BD		1.96	1	1.96	7.01	0.0226	
BE		0.0400	1	0.0400	0.1431	0.7124	
CD		74.39	1	74.39	266.22	<0.0001	
CE		5.50	1	5.50	19.68	0.0010	
DE		32.15	1	32.15	115.05	<0.0001	
A^2^		1.31	1	1.31	4.67	0.0435	
B^2^		1.31	1	1.31	4.67	0.047	
C^2^		1.31	1	1.31	4.67	0.0535	
D^2^		9.03	1	9.03	32.31	0.0001	
E^2^		1.31	1	1.31	4.67	0.0535	
Residual		3.07	11	0.2794			
Lack of Fit		3.07	6	0.5123		Not significant	
Pure Error		0.0000	5	0.0000			
Cor Total		577.76	31				
Std. Dev.	0.5286	R^2^	0.9947				
Mean	81.10	Adjusted R^2^	0.9850				
C.V. %	0.6518	Predicted R^2^	0.8594				
PRESS	81.25	Adeq Precision	44.6611				

Predictions were made using an ANN model to determine the biodiesel yield from LSO. The model had multiple input-single output structures. The experimental response from the design matrix provided the data to evaluate the network's ability to generalize. The data was divided into three sets: 70 % for training, 15 % for testing, and 15 % for validation. The study used a five-layered ANN structure with a hidden layer of ten neurons. The Levenberg Marquardt (trainlm) backpropagation method was used. The hidden layer used a tangent sigmoid transfer function (tansig), while the output layer used a linear transfer function (purelin). The system underwent a training process to minimize the discrepancy between expected and observed values for the hidden layer. This process involved using two to fifteen neurons and a trial-and-error approach. Increasing the number of hidden neurons increased the complexity of the network, resulting in fewer training data mistakes. The model's applicability and prediction capacity for linseed biodiesel catalyzed by CD-BaCl-IL were evaluated using the coefficient of determination (R^2^) and mean square error (MSE) correlation. The results, shown in Fig. 18, Fig. 19 indicated a high biodiesel production (R^2^ = 0.99, MSE = 0.27594). At an epoch value of 3, the high R^2^ value (0.99) and low MSE value suggested a good correlation between the experimental and predicted values. A lower MSE score [27,70,71] indicates an excellent model output.

**Fig. 18:** ANN regression graph for CD-BaCl-IL for LSO.

**Fig. 19:** MSE graph for CD-BaCl-IL for LSO.

The ANFIS structure that was built was utilised to forecast the generation of biodiesel using the CD-BaCl-IL catalyst, as depicted in Fig. 20. The membership function "trap mf" was chosen as the one with the lowest Mean Squared Error (MSE) among all the options, using a fixed number of 1000 epochs. The R-squared (R^2^) and the mean squared error (MSE) were utilised to assess the dependability of the network. The ANFIS model for linseed biodiesel catalyzed with CD-BaCl-IL has the following values: yield (R^2^- 0.9988, MSE-0.00038), as depicted in Fig. 19. The acquired R^2^ value of 0.99 indicates a high level of accuracy in predicting the process, which is supported by previous studies [31,72,73].

**Fig. 20:** The R^2^ ANFIS model prediction of linseed biodiesel catalyzed with CD-BaCl-IL.

### 3.10 Optimization process

The response variable, biodiesel yield, was optimised within the range of parameters studied in Table 11. The factors that yielded the highest biodiesel yield were a concentration of 2 wt%, a methanol/molar ratio of 6 mol/mol, a period of 1.5 h, a temperature of 50 °C, and an agitation speed of 400 rpm. These ideal values resulted in a predicted biodiesel yield of 97.097 %, as determined by a desire function of 1. The obtained yield closely corresponds to the experimental yield of 96.92 %, demonstrating a minimal discrepancy of 1.093 % between the experimental and anticipated values. The results compare favourably with the biodiesel yield of 97 % by Ullah et al. (2013) obtained at a catalyst concentration of 0.5 wt%, temperature (65 °C), 180 min reaction time and 6:1 methanol to oil molar ratio. This process confirms the correctness of the projected model and the dependability of the most effective combination [2,50,74].

#### 3.10.1 FT-IR analysis of the optimal biodiesel produced via heterogeneous catalyst

Fig. 21 displays the FT-IR analysis of the triglyceride of LSO methyl ester being converted to its optimum form using CD-BaCl-IL. The infrared (IR) peaks ranging from 1237 to 1744.4 cm^−1^ in LSO biodiesel are attributed to the bending vibrations of the O=C=O group. The IR spectra of the catalyst show two bands within the range of 2855.1–3008.0 cm^−1^ for linseed oil. These bands are attributed to the stretching of the C-H bonds in the alkyl group and the stretching of the C=O bonds in the esters group, respectively. Additionally, a peak at 1744.4 cm^−1^ is observed, which is also attributed to the C=O stretching of the esters group. The formation of these bands is a result of the triglyceride present in the oils that have not undergone conversion. The signal seen at 1159.2 cm^−1^ in LSO biodiesel corresponds to the presence of O-CH_3_, indicating the synthesis of methyl ester within the specified band range [75,76].

**Fig. 21:** FTIR analysis of optimal LSO biodiesel using CD-BaCl-IL catalyst.

#### 3.10.2 15: GC-MS analysis of the optimal biodiesel produced via heterogeneous catalyst

Fig. 22 depicts the transformation of a triglyceride of LSO into methyl ester using CDBaClIL. The graphic demonstrates the conversion of triglyceride into methyl esters. The highest peaks indicate the presence of methyl ester (18.011), while the lower peaks on the right side indicate the presence of monoglyceride (35.06), diglyceride (37.785), and unconverted triglyceride (41.971). This suggests that the triglycerides were successfully converted into biodiesel, resulting in a reduction in their levels to form biodiesel [37,77,78].

**Fig. 22:** GCMS analysis of optimal LSO biodiesel using CD-BaCl-IL catalyst.

Table 12 presents the physical and chemical properties of biodiesel made from linseed oil. This information is used to evaluate its competitiveness in comparison to normal diesel fuel. The biodiesel has a moisture content of 0.015 % and a specific gravity of 0.854, both of which are within an acceptable range. This suggests that the biodiesel is prone to spoiling. A iodine value of 3.12 indicates the process of converting unsaturated fatty acid triglycerides through transesterification. Furthermore, the biodiesel acid (3.2) and free fatty acid value (1.6) produced meet the ASTM specification for biodiesel, which protects the fuel from engine corrosion and deposits. Furthermore, biodiesel exhibits a reduced ignition delay time and improved flammability due to its increased cetane number. Engines face difficulties in starting and producing smoke when using fuels with low cetane levels. The biodiesel's cetane number in this instance, which is 49.9, exceeds the ASTM standard of 47. This implies that the biodiesel has lower emissions and undergoes a clean combustion process. These positive attributes can be ascribed to the specific catalyst used during the transesterification process. The aniline point, diesel index, flash point, cloud point, and gross calorific value of the linseed biodiesel were all determined to be within the specified ASTM criteria for biodiesel. In addition, the kinematic viscosity of the biodiesel, which is 5.5 mm^2^/s, compares favourably with the findings of Tariq et al. [46] value of 3.83 and Ullah et al. [79] value of 3.753 for linseed biodiesel, falls within the acceptable range set by the ASTM standards of 1.9–6.0. This indicates that the biodiesel can flow freely. This information is supported by Refs. [70,80,81]. The flash point of 172 compares favourably with the findings of Akram et al. [82] (161) and Ullah et al. [79] (177), on linseed biodiesel characterization via a base catalyst, they are within the minimal value of 130 as compared to the ASTM standard.

**Table 11:** Optimization process of LSO catalyzed by CD-BaCl-IL.

LSOcatalyzed by CDBaCLIL(RSM)	2	6	1.5	50	400	96.92	97.097

**Table 12:** Linseed biodiesel characterization.

Fuel properties	Biodiesel produced	ASTM D6751 standard
Free fatty acid value (mgKOH/g)	0.16	
Gross calorific value (J/g)	7855.32	
Diesel index	57.39	
API gravity	30.53	
Cetane number	49.9	min- 47
Iodine value (gI_2_/100 g)	3.12	
Flashpoint (^o^C)	172	min- 130
Kinematic viscosity @ 40°C (mm2s-1)	5.5	1.9–6.0
Specific gravity	0.854	
Cloud point (^o^C)	9.50	−15 to 15
Moisture (%)	0.015	
Aniline point (^o^F)	188.00	
Acid value (mg KOH/g)	0.32	Max 0.5

## 4 Conclusion

This study assessed the efficacy of RSM in predicting the transesterification of linseed oil utilising CD-BaCl-IL catalyst as a heterogeneous catalyst. The synthesized catalyst underwent characterization utilising a range of techniques, including FT-IR, SEM, XRF, XRD, and BET, to verify its activation for the transesterification process. The analysis of variance (ANOVA) validated that the process parameters had a substantial influence on the process. The transesterification process was evaluated using ANN and ANFIS models, which yielded successful results. The evaluation was based on statistical criteria such as R^2^ and MSE. The findings demonstrated that ANFIS exhibited superior performance compared to ANN in terms of process prediction. The data indicate that RSM successfully optimised the transesterification process of linseed biodiesel by decreasing process parameters, thereby providing a cost-efficient process. In addition, it was determined that the LHHW model could accurately describe the rate of transesterification. This model identifies the surface reaction between adsorbed triglyceride and alcohol as the rate-determining step. The rate constant exhibited a positive correlation with temperature, suggesting that the reaction was endothermic and took place at temperatures surpassing the boiling point of alcohol. The linseed oil biodiesel exhibited compliance with the parameters specified in the ASTM D6751 standards. Hence, the kinetic model that has been developed with the ideal parameters will be highly useful in the process of designing reactors for the manufacture of biodiesel. Further studies are recommended in developing nanocatalysts from clays and sourcing non-edible oils from the transesterification process.

## Data availability statement

Data will be made available on request.

## CRediT authorship contribution statement

**Kenechi Nwosu-Obieogu:** Writing – review & editing, Writing – original draft, Conceptualization. **Ude Callistus Nonso:** Resources, Methodology, Investigation. **Onukwuli Dominic Okechukwu:** Supervision. **Ezeugo Joseph:** Software, Resources, Project administration, Funding acquisition.

## Declaration of competing interest

The authors declare that they have no known competing financial interests or personal relationships that could have appeared to influence the work reported in this paper.
